The article "Network Pharmacology and Molecular Docking Analysis on the Pharmacological Mechanisms of Modified Sanmiaosan in Treating Ulcerative Colitis" was published in 2022. Journal: Comput Math Methods Med.

# Network Pharmacology and Molecular Docking Analysis on the Pharmacological Mechanisms of Modified Sanmiaosan in Treating Ulcerative Colitis

**DOI:** 10.1155/2022/2556521

**Published:** 2022-08-04

**Authors:** Yong Wang, Ying Sun, Ruoran Wang, Jisha Du, Qingqing Wang

**Affiliations:** ^1^School of Traditional Chinese Medicine, Shandong University of Traditional Chinese Medicine, Jinan 250355, China; ^2^Traditional Chinese Medicine Research Institute, Tai'an Hospital of Chinese Medicine, Tai'an 271000, China; ^3^Department of Neurosurgery, West China Hospital, Sichuan University, Chengdu 610000, China; ^4^Department of Nephrology, PLA Naval Medical Center, Shanghai 200052, China; ^5^Department of Neurology, PLA Naval Medical Center, Shanghai 200052, China

## Abstract

**Background:**

Modified Sanmiaosan is an effective cure in the treatment of ulcerative colitis, but its mechanisms of action remain unclear. This study revealed the pharmacological mechanisms of Modified Sanmiaosan acting on ulcerative colitis through a pharmacology approach.

**Materials and Methods:**

The active compounds and the targets of Modified Sanmiaosan were selected from the Traditional Chinese Medicine Systems Pharmacology database according to the absorption and metabolism. The UC-related therapeutic targets were collected from the PharmGKB database, the GeneCards database, the GADA database, and the OMIM database. The networks of “drug-component-target-disease” and “herbal-component-target” were constructed by the Cytoscape software. Protein–protein interaction network was generated by the STRING database. Gene Ontology (GO) and Kyoto Encyclopedia of Genes and Genomes (KEGG) pathway enrichment analyses were performed by the R software. Molecular docking technology was used to identify the affinity and activity between active compounds and targets.

**Results:**

The 80 effective ingredients of MSM were collected. A total of 5180 UC-related genes and the 153 key targets of MSM and UC-related were obtained. JUN, Akt1, and MAPK1 were identified as the “hub targets” involved in the effects of Modified Sanmiaosan on ulcerative colitis. Hub targets were mainly involved in inflammatory response and oxidative stress. As the results of GO analysis, biological processes such as DNA-binding transcription and RNA polymerization may participate in the treatment process; KEGG pathway analysis showed that hub targets were mainly involved in IL-17 signal pathway and TNF signal pathway of ulcerative colitis. The high affinity and activity of the active compounds and targets were verified through molecular docking.

**Conclusion:**

These findings demonstrate the active ingredients in Modified Sanmiaosan reduce inflammatory response by TNF and IL-17 signaling pathways to treat ulcerative colitis. Anti-inflammation and immune regulation may be the main mechanism of Modified Sanmiaosan in the treatment of ulcerative colitis. This study not only provide new insights into the development of a natural therapy for the prevention and treatment of ulcerative colitis but also proves a feasible method for discovering potential activated compounds from Chinese herbs.

The article "Network Pharmacology and Molecular Docking Analysis on the Pharmacological Mechanisms of Modified Sanmiaosan in Treating Ulcerative Colitis" was published in 2022. Journal: Comput Math Methods Med.

## 1. Introduction

Ulcerative colitis (UC) is an idiopathic, chronic inflammatory disorder of the colonic mucosa, which starts in the rectum and progresses proximally in a continuous manner through the entire colon. It is characterized by chronic mucosal inflammation that recurs for life. The most prominent symptoms include hematochezia, diarrhea, and abdominal pain. Moreover, several patients with UC are affected by extraintestinal complications. The incidence and burden of UC are on the rise globally. The annual incidence of UC is between 8 and 14 cases per 100,000 persons in the Western population, and the prevalence is increasing in Asia [1, 2]. First-line therapy includes 5-aminosalicylic acid and corticosteroids. Glucocorticoids and biological agents can be added when 5-aminosalicylic acid therapy is ineffective [2]. Because of the marked side effects of Western medicine, patients still have difficulty adhering to treatment, leading to the discontinuation of therapy. As an important component of complementary and alternative medicine, traditional Chinese medicine (TCM) has been widely used to treat and prevent UC and has shown significant positive effects and low recurrence rates [3].

In TCM, clearing heat and removing dampness is a key method for UC treatment [4]. Sanmiao powder is a classic TCM prescription for clearing heat and drying dampness, including *Atractylodes lancea*, *Phellodendri chinensis*, and *Radix Achyranthis bidentatae* [5].

Based on the formulation of Sanmiaosan, *Bletilla striata* and *Agrimonia eupatoria* were added to form Modified Sanmiaosan (MSM). MSM has been reported to have achieved a good curative effect in the treatment of UC [6]. *Atractylodes lancea* has proven regulation of the nuclear factor *κ*B (NF-*κ*B) signaling pathway to reduce lipopolysaccharide-induced inflammatory injury of human colonic epithelial cells [7]. *Agrimonia eupatoria* ameliorates dextran sodium sulfate-induced colitis through NF-*κ*B signaling pathway [8]. *Bletilla striata* effectively inhibited the release of intestinal inflammatory cytokines such as IL-6, TNF-*α*, and IL-1*β* and attenuated dysfunction of the intestinal barrier in UC mouse model induced by 3% dextran sodium sulfate [9]. MSM is effective in the treatment of UC, but its underlying pharmacological properties and mechanisms of action remain unclear [6].

The article "Network Pharmacology and Molecular Docking Analysis on the Pharmacological Mechanisms of Modified Sanmiaosan in Treating Ulcerative Colitis" was published in 2022. Journal: Comput Math Methods Med.

Network pharmacology is an innovative way to explore new drug targets, which can identify active drug ingredients by investigating the relationship between drug components and disease targets. Based on the intersection of drug targets with key genes, the drug-target network can be constructed, and the potential mechanism can be explored. This method can be helpful to discern the pharmacological action and mechanism of TCM [10]. In this study, we adopted a network pharmacology approach to investigate how MSM exerts therapeutic effects on UC by target prediction, biological function, and pathway analysis. This study may provide a useful reference for the identification of the therapeutic mechanisms of TCM.

## 2. Materials and Methods

### 2.1. MSM Ingredients

The components of MSM (*Atractylodes lancea*, *Phellodendri chinensis*, *Radix Achyranthis bidentatae*, *Bletilla striata*, *Agrimonia eupatoria*) were searched in the Traditional Chinese Medicine Systems Pharmacology (TCMSP) database (https://old.tcmsp-e.com/tcmsp.php/) by the ADME model. The ingredients with OB ≥ 30% and DL ≥ 0.18 were selected. OB represents the ability of a compound to circulate in the body after oral administration. DL is an indicator for determining the similarity of physicochemical properties of a compound with conventional drugs. The target names of all compounds were transformed into UniProt IDs using the UniProt database (http://www.uniprot.org/).

### 2.2. Databases to Identify and Predict the Targets of UC

By searching the keywords “Ulcerative colitis”, the targets related to UC were collected from the GeneCards database (https://www.genecards.org), the OMIM database (https://omim.org), the PharmGKB database (https://www.pharmgkb.org), and the Genetic Association Database (GADA, https://www.Geneticassociationdb.nih.gov) [11].

### 2.3. Key Targets

The Venn diagram generation software Venny 2.1 was used to identify potential key targets of MSM in treating UC.

### 2.4. Construction of Network Relationships

The “drug-component-target-disease” and “herbal-component-target” networks were constructed for visualization using Cytoscape version 3.6.1 (http://www.cytoscape.org/). The nodes in the network represent herbs, chemicals, and potential targets; the edges indicate interactions between them. In the network, the quantity of each edge was defined as “degree.”

### 2.5. Protein-Protein Interactions (PPI)

Key targets were imported into the STRING (https://string-db.org/) database to build the PPI network model. The minimum required interaction score was set as “medium confidence = 0.9,” while the other parameters remain as default. In the network, the size of the nodes represents the degree size. The higher the degree, the better the correlation between the proteins. Targets with scores in the top 30 were selected as core targets [12].

The article "Network Pharmacology and Molecular Docking Analysis on the Pharmacological Mechanisms of Modified Sanmiaosan in Treating Ulcerative Colitis" was published in 2022. Journal: Comput Math Methods Med.

### 2.6. Enrichment Analysis

Gene Ontology (GO) enrichment analysis and Kyoto Encyclopedia of Genes and Genomes (KEGG) pathway analysis of target genes were performed using the R software (version 3.6.0); the *p* value was defined as <0.05 and *Q* < 0.05. The top 20 enriched pathways of GO and KEGG were reported as bubble charts and bar graphs [12].

### 2.7. Molecular Docking Analysis

Download the SDF format of 3D structure of kaempferol, luteolin, and quercetin in PubChem, and then import it into ChemDraw 3D. Use the MM 2 module to minimize the energy, obtain the optimal conformation of the lowest energy, and save it as a mol 2 file. MAPK1, AKT1, and JUN were retrieved from the PDB database to obtain the protein structure; their PDB IDs are 6slg, 7nh5, and 1a02. Then, PyMOL is used for visualization. MGTools 1.5.6 is used for water removal, hydrogenation, charge calculation, and nonpolar hydrogen combination. Then, use AutoDock Vina 1.1 2 for docking the ligand with the receptor [13].

## 3. Results

### 3.1. Distribution of MSM Ingredients

80 ingredients of MSM that satisfied the DL criteria were retrieved from the TCMSP database, including 9 *Atractylodes lancea* ingredients, 37 *Phellodendri chinensis* ingredients, 20 *Radix Achyranthis bidentatae* ingredients, 9 *Bletilla striata* ingredients, and 5 *Agrimonia eupatoria* ingredients (Table 1).

### 3.2. Potential Targets of MSM in Treating UC

The targets of active ingredients were downloaded from the TCMSP database. A total of 1458 UC-related targets were obtained from the GADA database, 15 UC-related targets were obtained from the PharmGKB database, 4800 UC-related targets were obtained from the GeneCards database, and 7 were obtained from the OMIM database. A total of 5180 UC-related targets were retrieved after eliminating the duplicate entries. The MSM targets and UC targets were intersected to obtain 153 targets, which were noted as “key targets” to construct the PPI network and for GO\KEGG analysis (Figure 1).

### 3.3. Analysis of “Drug-Component-Target-Disease” Network and “Herbal-Component-Target” Network

The “drug-component-disease-target” network consisted of 80 active ingredients and 153 key targets. In Figure 2(a), the purple oval represents UC, the pink polygon represents MSM, the green diamond represents the active ingredient of MSM, and the blue rectangle represents the disease targets corresponding to the active ingredients of the drug. There are 192 nodes and 996 edges in the drug-component-disease-target network. The three active components with the highest “degree” values are quercetin, kaempferol, and luteolin (as shown in Table 2); it is suggested that it is the key active ingredient of the network. In the herbal-component-target network (Figure 2(b)), the blue rectangle nodes represent the targets.

The article "Network Pharmacology and Molecular Docking Analysis on the Pharmacological Mechanisms of Modified Sanmiaosan in Treating Ulcerative Colitis" was published in 2022. Journal: Comput Math Methods Med.

### 3.4. PPI Network Construction and PPI-Based Hub Target Identification

The 153 key targets were uploaded to the STRING database (https://string-db.org/cgi/input.pl) to construct the PPI network. In Figure 3, there were 153 nodes and 547 edges in the PPI network (PPI enrichment *p* value: < 1.0*e*-16), which reflects the complexity of the disease mechanism and the characteristics of TCM for disease treatment. Gene targets with a high degree in the PPI network include JUN, Akt1, and mitogen-activated protein kinase-1 (MAPK1); these genes were considered “hub targets” involved in the effects of MSM on UC (Figures 3 and 4).

### 3.5. GO and KEGG Enrichment Analyses

153 key targets were selected for GO and KEGG pathway enrichment analyses. The top 20 GO analysis results are shown in Figures 5(a) and 5(b). The GO enrichment analysis reported that the top results are chiefly involved in DNA-binding transcription activator activity, RNA polymerase II-specific, cytokine receptor binding, transcription factor activity, RNA polymerase II proximal, promoter sequence-specific DNA binding, protein serine/threonine kinase activity, receptor ligand activity, and cytokine activity.

The top 20 pathways are shown in Figures 6(a) and 6(b). Pathways unrelated to UC were excluded. The KEGG pathway analysis showed these targets to be mainly associated with IL-17 and TNF signaling pathways of UC (Figures 7(a) and 7(b)).

Active compounds from MSM could target multiple proteins and subsequently initiate complex signal transduction, regulate inflammation-related pathways, restrain the progression of UC, and provide a better prognosis in patients.

### 3.6. Molecular Docking Studies to Evaluate Interactions between MSM and UC Targets

The top three targets (JUN, Akt1, and MAPK1) in the PPI network and the top three active ingredients (quercetin, kaempferol, and luteolin) in the network were selected for molecular docking. Molecular docking showed that quercetin, kaempferol, and luteolin can closely bind three targets (JUN, Akt1, and MAPK1).  Table 3 shows the energy docking scores. The lower the binding energy between small molecule ligands and protein receptors, the better the affinity between them and the more stable the concept. It is generally accepted that binding energy which is less than −4.25 kcal/mol, −5.0 kcal/mol, or−7.0 kcal/mol indicates a certain, good, or strong binding activity between the ligand and the receptor, respectively [13].

The article "Network Pharmacology and Molecular Docking Analysis on the Pharmacological Mechanisms of Modified Sanmiaosan in Treating Ulcerative Colitis" was published in 2022. Journal: Comput Math Methods Med.

The PyMOL software was used for visual analysis of molecular docking. The 3D structures of JUN, Akt1, and MAPK1 are shown in Figures 8(a)–8(c). We selected the top three receptor proteins with the lowest energy value and the ligand that bound to these receptor proteins for visualization (see Figures 9(a)–9(c)). It shows the best docking combinations for Akt1 and the compound, including kaempferol, luteolin, and quercetin, with binding energies of –9.2, –9.8, and –10.1 kcal/mol, respectively. It indicates that there is strong binding activity between receptor and ligand.

## 4. Discussion

In this study, network pharmacology methods were used to explore the potential targets and mechanisms of MSM in treating UC. A total of 80 active compounds were identified using the TCMSP database (OB ≥ 30% and DL ≥ 0.18) and 5180 UC-related targets were obtained from the PharmGKB database, the GeneCards database, the GADA database, and the OMIM database. The MSM targets and UC targets were intersected by using a Venn tool to obtain 153 targets, identified as “key targets” for PPI network construction and GO\KEGG analysis. The PPI network was constructed by uploading these 153 key targets to the STRING database. Targets with high degree value in the PPI network included JUN, Akt1, and MAPK1; these genes were considered “hub targets” involved in the effects of MSM on UC. GO and KEGG enrichment analyses of the 153 key targets revealed that IL-17 and TNF signaling pathways were the most enriched pathways. Cytoscape was used to generate the network showing the relationship between drug components and targets containing 80 active ingredients and 153 key targets. The treatment of diseases by TCM was mainly achieved by the synergistic action of many active compounds on multiple targets. Network pharmacology was used to reveal the underlying mechanisms with the above characteristics.

### 4.1. Active Ingredients of MSM

As previously reported, 153 active compounds of MSM in the treatment of UC were obtained. Through network analysis, the most promising compounds were identified as quercetin, kaempferol, luteolin, *β*-sitosterol, and baicalein. This finding suggests that these compounds may be important for the therapeutic role of MSM in UC and warrant further investigation. As reported, quercetin is a polyphenolic flavonoid compound whose antioxidant activity has been investigated in numerous studies. It is effective in treating and preventing various diseases due to its effect on glutathione, enzyme activity, signal transduction pathways, and reactive oxygen species (ROS) production [14]. Kaempferol is one of the most common polyphenols attached to sugar groups in fruits and vegetables [15]. Kaempferol is a proven regulator of ER stress and autophagy and exhibits protective effects on malfunctioning cells [16]. In a novel epithelial-endothelial cell coculture model, kaempferol is confirmed to reduce lipopolysaccharide- (LPS-) induced IL-8 secretion and barrier dysfunction of Caco-2 cells [17]. Luteolin is a flavonoid found in plants, with anticancer activity against various types of human malignancies [18]. Moreover, luteolin modulates many inflammatory pathways by suppressing proinflammatory mediators (interleukin- (IL-) 1*β*, IL-6, IL-17, IL-22, and TNF-*α*) and regulates various inflammation-related signaling pathways [19]. *β*-Sitosterol is a bioactive compound found in the plant cell membrane, with a chemical structure similar to cholesterol. *β*-Sitosterol is known to possess various benefit actions such as immunomodulatory effect, anticancer, and anti-inflammatory activity [20]. Various studies have demonstrated the antioxidative, anti-inflammatory, and antitumor activities of baicalein. Baicalein has also been reported to ameliorate dextran sulfate sodium-induced colitis by inhibiting NF-*κ*B and STAT3 signaling pathways and mitigating radiation-induced enteritis by improving endothelial dysfunction, thereby preventing the development of colitis-associated cancer [21, 22].

The article "Network Pharmacology and Molecular Docking Analysis on the Pharmacological Mechanisms of Modified Sanmiaosan in Treating Ulcerative Colitis" was published in 2022. Journal: Comput Math Methods Med.

### 4.2. Core Targets of MSM in UC

PPI network identified JUN, Akt1, and MAPK1 as core targets. These targets involved in inflammation, apoptosis, and other processes may play an important role in the therapeutic effect of MSM in UC. JUN is a major component of the heterodimeric transcription factor AP-1 and a critical driver of cell proliferation and apoptosis [23]. Additionally, various growth factors, cytokines, and stress stimulate the activation of c-Jun and then regulate biological processes [24]. Akt1 is one of the serine/threonine protein kinases called Akt kinase, which is integral for insulin signaling, endothelial function, and metabolic regulation [25]. Akt plays an important role as a protumorigenic and metastatic regulator in cancer due to its specific effects on cancer cells, tumor endothelial cells, and stromal cells [26]. AKT1 has been demonstrated to be involved in cell survival, and proliferation, and as a downstream factor of PI3K. MAPK is an interconnected signaling cascade with involvement in cell growth, differentiation, inflammatory response, and other important cellular, physiological, and pathological pathways [27]. The regulation of PI3K/Akt and MAPK/Akt pathways by MSM may play an important role in its therapeutic effect in UC. The results of molecular docking studies showed that quercetin, kaempferol, and luteolin can closely bind three targets (JUN, Akt1, and MAPK1).

The article "Network Pharmacology and Molecular Docking Analysis on the Pharmacological Mechanisms of Modified Sanmiaosan in Treating Ulcerative Colitis" was published in 2022. Journal: Comput Math Methods Med.

### 4.3. MSM Pathways in Treating UC

We performed GO enrichment analysis and KEGG enrichment analysis of the 153 potential targets. GO analysis results showed that biological processes such as DNA-binding transcription activator activity, RNA polymerase II-specific cytokine receptor binding, transcription factor activity, RNA polymerase II proximal, promotor sequence-specific DNA binding, protein serine/threonine kinase activity, receptor ligand activity, and cytokine activity may play a role in the treatment of UC. KEGG pathway analysis showed that these targets were mainly involved in IL-17 and TNF signaling pathways of UC.

The pathogenesis of UC consists of immuno-inflammatory pathways, including the epithelial barrier, commensal microflora, dysregulation of immunological responses, and leukocyte recruitment.

Proinflammatory cytokines (tumor necrosis factor-*α* (TNF-*α*), IL-1, IL-6, IL-9, IL-13, and IL-33) play a significant role in upregulation, while anti-inflammatory cytokines (transforming growth factor-*β*, IL-10, and IL-37) play a significant role in downregulation of disease progression. The imbalance of proinflammatory and anti-inflammatory cytokines is a key factor in the immune dysfunction of intestinal mucosal [28]. A clearer understanding of the inflammatory pathways of UC regulation by MSM may aid in the development of drug screening.

The proinflammatory cytokines IL-17 have been implicated in the pathogenesis of inflammatory bowel disease and have received a lot of attention for their activity. IL-17 signaling can induce a cascade of proinflammatory molecules such as TNF, IFN*γ*, IL-22, lymphotoxin, IL-1*β*, and LPS [29]. TNF signaling pathways play a vital role in the typical immune response by regulating several downstream processes [30]. The IL-17 and TNF signaling pathways are considered classical signaling pathways in immune reaction. These two signaling pathways can activate the intracellular molecular signal, leading to the activation of cells in the ER, which results in inflammation of intestinal mucosal cells [28]. As biological response modifiers, antibodies neutralizing TNF-*α* have been used in studies and clinical practice [31].

In conclusion, chronic inflammation, the main pathological process of UC, may lead to the accumulation of high levels of proinflammatory cytokines within the colonic mucosa and could lead to cancer. The risk of colorectal cancer (CRC) in patients with UC is 2.4-fold higher compared to the general population [2]. Improving inflammatory response is a viable approach for the treatment of UC and prevention of cancer. This study showed that MSM improved the inflammatory response of UC via the IL-17 and TNF signaling pathways, which may prove beneficial to alleviate symptoms and prevent cancer. The results of molecular docking studies showed that the compound (quercetin, kaempferol, and luteolin) can closely bind the core targets (JUN, Akt1, and MAPK1) [32].

The article "Network Pharmacology and Molecular Docking Analysis on the Pharmacological Mechanisms of Modified Sanmiaosan in Treating Ulcerative Colitis" was published in 2022. Journal: Comput Math Methods Med.

However, this study has limitations. The mechanism of MSM in the treatment of UC through the IL-17 and TNF signaling pathways needs to be further explored. In addition, the mechanism of MSM determined in this study needs to be further analyzed and verified through experimental research. We will further use molecular biology methods to investigate the effects and molecular mechanism of MSM in treating UC and conduct random clinical trials to identify the effectiveness of MSM in patients with UC.

## Figures and Tables

**Figure 1:** Venn diagram of the targets of the active ingredients of the drug and the disease-related targets.

**Figure 2:** (a) “Drug-component-target-disease” network construction. The blue rectangle nodes represent the targets; the green diamond nodes represent ingredients of MSM. (b) “Herbal-component-target” network construction. The blue rectangle nodes represent the targets.

**Figure 3:** PPI network of the core targets.

**Figure 4:** 30 core targets determined in the PPI network.

**Figure 5:** (a) Dot plot of GO enrichment analysis. The “*x*” coordinate indicates the number of enriched genes, and the color of the dot represents the *p* value of the corresponding term. The larger the dot, the more genes are enriched. (b) Bar plot of GO enrichment analysis.

**Figure 6:** (a) Dot plot of KEGG enrichment analysis. The size of the bubble represents the number of targets enriched in the indicated pathway, and the color of the bubble represents the *p* value of enrichment. (b) Bar plot of KEGG enrichment analysis.

**Figure 7:** (a) TNF pathway map of MSM for their potential treatment of UC. Nodes in red represent MSM-UC-related target. (b) IL-17 pathway map of MSM for their potential treatment of UC. Nodes in red represent MSM-UC-related target.

**Figure 8:** (a) The 3D structures of JUN. (b) The 3D structures of Akt1. (c) The 3D structures of MAPK1.

**Figure 9:** (a) Schematic diagram of the docking of AKT1 and kaempferol. (b) Schematic diagram of the docking of AKT1 and luteolin. (c) Schematic diagram of the docking of AKT1 and quercetin.

**Table 1:** Active ingredients of MSM.

Herbal	Mol ID	Molecule name	OB	DL
AE	MOL000006	Luteolin	36.16	0.25
AE	MOL000422	Kaempferol	41.88	0.24
AE	MOL001002	Ellagic acid	43.06	0.43
AE	MOL000098	Quercetin	46.43	0.28
AE	MOL000492	(+)-Catechin	54.83	0.24
RAB	MOL001006	Poriferasta-7,22E-dien-3beta-ol	42.98	0.76
RAB	MOL012461	28-Norolean-17-en-3-ol	35.93	0.78
RAB	MOL012505	Bidentatoside,ii_qt	31.76	0.59
RAB	MOL012537	Spinoside A	41.75	0.4
RAB	MOL012542	*β*-Ecdysterone	44.23	0.82
RAB	MOL001454	Berberine	36.86	0.78
RAB	MOL001458	Coptisine	30.67	0.86
RAB	MOL000173	Wogonin	30.68	0.23
RAB	MOL002643	Delta 7-stigmastenol	37.42	0.75
RAB	MOL002714	Baicalein	33.52	0.21
RAB	MOL002776	Baicalin	40.12	0.75
RAB	MOL002897	Epiberberine	43.09	0.78
RAB	MOL000358	Beta-sitosterol	36.91	0.75
RAB	MOL003847	Inophyllum E	38.81	0.85
RAB	MOL000422	Kaempferol	41.88	0.24
RAB	MOL004355	Spinasterol	42.98	0.76
RAB	MOL000449	Stigmasterol	43.83	0.76
RAB	MOL000785	Palmatine	64.6	0.65
RAB	MOL000085	Beta-daucosterol_qt	36.91	0.75
RAB	MOL000098	Quercetin	46.43	0.28
BS	MOL005755	1-(4-Hydroxybenzyl)-4-methoxy-9,10-dihydrophenanthrene-2,7-diol	54.18	0.55
BS	MOL005756	2,3,4,7-Tetramethoxyphenanthrene	39.09	0.29
BS	MOL005759	2,7-Dihydroxy-4-methoxyphenanthrene-2,7-O-diglucoside	30.22	0.74
BS	MOL005761	3-(p-Hydroxybenzyl)-4-methoxy-9,10-dihydrophenanthrene	37.98	0.55
BS	MOL005766	3,7-Dihydroxy-2,4-dimethoxyphenanthrene-3-O-glucoside	31.46	0.78
BS	MOL005768	4,7-Dihydroxy-1-p-hydroxybenzyl-2-methoxy-9,10-dihydrophenanthrene	30.54	0.55
BS	MOL005770	Bletlol A	54.43	0.55
BS	MOL005773	Blespirol	43.74	0.86
BS	MOL005776	1-(2,7-Dihydroxy-4-methoxy-1-phenanthryl)-4-methoxyphenanthrene-2,7-diol	35.22	0.67
AL	MOL000173	Wogonin	30.68	0.23
AL	MOL000179	2-Hydroxyisoxypropyl-3-hydroxy-7-isopentene-2,3-dihydrobenzofuran-5-carboxylic	45.2	0.2
AL	MOL000184	NSC63551	39.25	0.76
AL	MOL000186	Stigmasterol 3-O-beta-D-glucopyranoside_qt	43.83	0.76
AL	MOL000188	3*β*-Acetoxyatractylone	40.57	0.22
AL	MOL000085	Beta-daucosterol_qt	36.91	0.75
AL	MOL000088	Beta-sitosterol 3-O-glucoside_qt	36.91	0.75
AL	MOL000092	Daucosterin_qt	36.91	0.76
AL	MOL000094	Daucosterol_qt	36.91	0.76
PC	MOL001454	Berberine	36.86	0.78
PC	MOL001458	Coptisine	30.67	0.86
PC	MOL002636	Kihadalactone A	34.21	0.82
PC	MOL013352	Obacunone	43.29	0.77
PC	MOL002641	Phellavin_qt	35.86	0.44
PC	MOL002643	Delta 7-stigmastenol	37.42	0.75
PC	MOL002644	Phellopterin	40.19	0.28
PC	MOL002651	Dehydrotanshinone II A	43.76	0.4
PC	MOL002652	delta7-Dehydrosophoramine	54.45	0.25
PC	MOL002656	Dihydroniloticin	36.43	0.81
PC	MOL002659	Kihadanin A	31.6	0.7
PC	MOL002660	Niloticin	41.41	0.82
PC	MOL002662	Rutaecarpine	40.3	0.6
PC	MOL002663	Skimmianin	40.14	0.2
PC	MOL002666	Chelerythrine	34.18	0.78
PC	MOL000449	Stigmasterol	43.83	0.76
PC	MOL002668	Worenine	45.83	0.87
PC	MOL002670	Cavidine	35.64	0.81
PC	MOL002671	Candletoxin A	31.81	0.69
PC	MOL002672	Hericenone H	39	0.63
PC	MOL002673	Hispidone	36.18	0.83
PC	MOL000358	Beta-sitosterol	36.91	0.75
PC	MOL000622	Magnograndiolide	63.71	0.19
PC	MOL000762	Palmidin A	35.36	0.65
PC	MOL000785	Palmatine	64.6	0.65
PC	MOL000787	Fumarine	59.26	0.83
PC	MOL000790	Isocorypalmine	35.77	0.59
PC	MOL000098	Quercetin	46.43	0.28
PC	MOL001131	Phellamurin_qt	56.6	0.39
PC	MOL001455	(S)-Canadine	53.83	0.77
PC	MOL001771	Poriferast-5-en-3beta-ol	36.91	0.75
PC	MOL002894	Berberrubine	35.74	0.73
PC	MOL005438	Campesterol	37.58	0.71
PC	MOL006392	Dihydroniloticin	36.43	0.82
PC	MOL006401	Melianone	40.53	0.78
PC	MOL006413	Phellochin	35.41	0.82
PC	MOL006422	Thalifendine	44.41	0.73

AL: *Atractylodes lancea*; PC: *Phellodendri chinensis*; RAB: *Radix Achyranthis bidentatae*; BS: *Bletilla striata*; AE: *Agrimonia eupatoria*.

The article "Network Pharmacology and Molecular Docking Analysis on the Pharmacological Mechanisms of Modified Sanmiaosan in Treating Ulcerative Colitis" was published in 2022. Journal: Comput Math Methods Med.

**Table 2:** The degree of active ingredients of MSM.

Active ingredients	Degree
Kaempferol	75
Luteolin	46
Quercetin	340

**Table 3:** Energy docking scores (kcal mol^−1^).

	Kaempferol	Luteolin	Quercetin
MAKP1	-8.1	-8	-8
AKT1	-9.2	-9.8	-10.1
JUN	-6.5	-6.6	-6.6

## Data Availability

The datasets used during the current study are available from the corresponding author on reasonable request.

## References

[1] Burisch J., Jess T., Martinato M., Lakatos P. L. (2013). The burden of inflammatory bowel disease in Europe. *Journal of Crohn's and Colitis*.

[2] Rivera A. P., Monar G. V. F., Islam H. (2022). Ulcerative colitis-induced colorectal carcinoma: a deleterious concatenation. *Cureus*.

[3] Si-Yu C. A. O., Sheng-Jie Y. E., Wei-Wei W. A. N. G., Bing W. A. N. G., Zhang T., Yi-Qiong P. U. (2019). Progress in active compounds effective on ulcerative colitis from Chinese medicines. *Chinese Journal of Natural Medicines*.

[4] Ning L. (2018). *The Clinical Efficacy and Data Minging of Professor Xu Jing-Fan Prescripyion for Treating Ulcerative Colitis*.

[5] Qian H., Jin Q., Liu Y. (2020). Study on the multitarget mechanism of Sanmiao pill on gouty arthritis based on network pharmacology. *Evidence-Based Complementary and Alternative Medicine*.

[6] Wang K., Guo J., Chang X., Gui S. (2022). Painong-San extract alleviates dextran sulfate sodium-induced colitis in mice by modulating gut microbiota, restoring intestinal barrier function and attenuating TLR4/NF-*κ*B signaling cascades. *Journal of Pharmaceutical and Biomedical Analysis*.

[7] Yu Y., Wu Z., Han Y. (2021). Comparison of the effects of essential oil obtained from the crude and bran- processed Atractylodes lancea on lipopolysaccharide-induced inflammatory injury of human colonic epithelial cells by downregulating the IKK/NF-*κ*B signaling pathway. *Evidence-Based Complementary and Alternative Medicine*.

The article "Network Pharmacology and Molecular Docking Analysis on the Pharmacological Mechanisms of Modified Sanmiaosan in Treating Ulcerative Colitis" was published in 2022. Journal: Comput Math Methods Med.

[8] Li C., Wang M., Sui J., Zhou Y., Chen W. (2021). Protective mechanisms of Agrimonia pilosa Ledeb in dextran sodium sulfate-induced colitis as determined by a network pharmacology approach. *Acta Biochimica et Biophysica Sinica*.

[9] Zhu T., Hu B., Ye C. (2022). Bletilla striata oligosaccharides improve ulcerative colitis by regulating gut microbiota and intestinal metabolites in dextran sulfate sodium-induced mice. *Frontiers in Pharmacology*.

[10] Wang K., Lei L., Cao J. (2021). Network pharmacology-based prediction of the active compounds and mechanism of Buyang Huanwu decoction for ischemic stroke. *Experimental and Therapeutic Medicine*.

[11] Hu W., Fu W., Wei X., Yang Y., Lu C., Liu Z. (2019). A network pharmacology study on the active ingredients and potential targets of Tripterygium wilfordii hook for treatment of rheumatoid arthritis. *Evidence-based Complementary and Alternative Medicine*.

[12] Qin L., Chen H., Ding X. (2021). Utilizing network pharmacology to explore potential mechanisms of YiSui Nong Jian formula in treating myelodysplastic syndrome. *Bioengineered*.

[13] Liu J., Liu J., Tong X. (2021). Network pharmacology prediction and molecular docking-based strategy to discover the potential pharmacological mechanism of Huai Hua San against ulcerative colitis. *Drug Design, Development and Therapy*.

[14] Xu D., Hu M. J., Wang Y. Q., Cui Y. L. (2019). Antioxidant activities of quercetin and its complexes for medicinal application. *Molecules*.

[15] Dabeek W. M., Marra M. V. (2019). Dietary quercetin and kaempferol: bioavailability and potential cardiovascular-related bioactivity in humans. *Nutrients*.

[16] Ashrafizadeh M., Tavakol S., Ahmadi Z., Roomiani S., Mohammadinejad R., Samarghandian S. (2020). Therapeutic effects of kaempferol affecting autophagy and endoplasmic reticulum stress. *Phytotherapy Research*.

[17] Bian Y., Dong Y., Sun J. (2020). Protective effect of kaempferol on LPS-induced inflammation and barrier dysfunction in a coculture model of intestinal epithelial cells and intestinal microvascular endothelial cells. *Journal of Agricultural and Food Chemistry*.

[18] Imran M., Rauf A., Abu-Izneid T. (2019). Luteolin, a flavonoid, as an anticancer agent: a review. *Biomedicine & Pharmacotherapy*.

[19] Gendrisch F., Esser P. R., Schempp C. M., Wölfle U. (2021). Luteolin as a modulator of skin aging and inflammation. *Biofactors*.

[20] Babu S., Jayaraman S. (2020). An update on *β*-sitosterol: a potential herbal nutraceutical for diabetic management. *Biomedicine & Pharmacotherapy*.

[21] Zhong X., Surh Y. J., Do S. G. (2019). Baicalein inhibits dextran sulfate sodium-induced mouse colitis. *Journal of Cancer Prevention*.

The article "Network Pharmacology and Molecular Docking Analysis on the Pharmacological Mechanisms of Modified Sanmiaosan in Treating Ulcerative Colitis" was published in 2022. Journal: Comput Math Methods Med.

[22] Jang H., Lee J., Park S. (2019). Baicalein mitigates radiation-induced enteritis by improving endothelial dysfunction. *Frontiers in Pharmacology*.

[23] Griffin M. F., Borrelli M. R., Garcia J. T. (2021). JUN promotes hypertrophic skin scarring via CD36 in preclinical in vitro and in vivo models. *Science Translational Medicine*.

[24] Yu W., Wang B., Zhou L., Xu G. (2021). Endoplasmic reticulum stress-mediated p62 downregulation inhibits apoptosis via c-jun upregulation. *Biomolecules & Therapeutics*.

[25] Alwhaibi A., Verma A., Adil M. S., Somanath P. R. (2019). The unconventional role of Akt 1 in the advanced cancers and in diabetes-promoted carcinogenesis. *Pharmacological Research*.

[26] Alwhaibi A., Verma A., Adil M. S., Somanath P. R. (2019). The unconventional role of Akt1 in the advanced cancers and in diabetes- promoted carcinogenesis. *Pharmacological Research*.

[27] Braicu C., Buse M., Busuioc C. (2019). A comprehensive review on MAPK: a promising therapeutic target in cancer. *Cancers (Basel)*.

[28] Tatiya-Aphiradee N., Chatuphonprasert W., Jarukamjorn K. (2018). Immune response and inflammatory pathway of ulcerative colitis. *Journal of Basic and Clinical Physiology and Pharmacology*.

[29] Schmitt H., Neurath M. F., Atreya R. (2021). Role of the IL23/IL17 pathway in Crohn’s disease. *Frontiers in Immunology*.

[30] Holbrook J., Lara-Reyna S., Jarosz-Griffiths H., McDermott M. F. (2019). Tumour necrosis factor signalling in health and disease. *F1000Research*.

[31] Li Y., Chen J., Bolinger A. A. (2021). Target-based small molecule drug discovery towards novel therapeutics for inflammatory bowel diseases. *Inflammatory Bowel Diseases*.

[32] Zhang L., Han L., Wang X. (2021). Exploring the mechanisms underlying the therapeutic effect of Salvia miltiorrhiza in diabetic nephropathy using network pharmacology and molecular docking. *Bioscience Reports*.

